This article has been retracted.

# Community Wellbeing Under China-Pakistan Economic Corridor: Role of Social, Economic, Cultural, and Educational Factors in Improving Residents’ Quality of Life

**DOI:** 10.3389/fpsyg.2021.816592

**Published:** 2022-03-25

**Authors:** Jaffar Aman, Jaffar Abbas, Guoqing Shi, Noor Ul Ain, Likun Gu

**Affiliations:** ^1^Postdoctoral Station, School of Public Administration and Sociology, Hohai University, Nanjing, China; ^2^School of Media and Communication, Shanghai Jiao Tong University, Shanghai, China; ^3^Antai College of Economics and Management, Shanghai Jiao Tong University, Shanghai, China; ^4^School of Management Sciences, Quad-i-Azam University, Islamabad, Pakistan; ^5^School of Public Administration, Asian Research Center, Hohai University, Nanjing, China

**Keywords:** COVID-19, safety, environment risks, regional development, community mental wellbeing, educational opportunities

## Abstract

This present article explores the effects of cultural value, economic prosperity, and community mental wellbeing through multi-sectoral infrastructure growth projects under the Belt and Road Initiative. The implications of the social exchange theory are applied to observe the support of the local community for the China-Pakistan Economic Corridor (CPEC). This study explores the CPEC initiative, it’s direct social, cultural, economic development, and risk of environmental factors that affect residents’ lives and the local community’s wellbeing. CPEC is a multibillion-dollar project to uplift economic growth and free trade between Pakistan, China, and other regional stakeholders. Although CPEC is still in its initial phases with partial startups, policymakers and government officials claim this mega project as a “game-changer” in the region, mainly for Pakistan and China. This gigantic project offers the significant potential to generate business slews and employment opportunities with international outreach. Due to the term’s newness, numerous studies have recently explored the macro and microeconomic benefits of the CPEC initiatives; still, these projects are theoretical. The existing literature insufficiently explored how helpful CPEC would be to a specific group and how residents perceive its advantages. This study fills in the literature gaps and explores the likely advantageous potential of the CPEC for the regional states. The study applied a convenient sampling technique for the data collection process. It used a mixed-method approach to gain scientific results, with a standardized questionnaire survey of 459 people (300 men and 159 women) from five major cities of Pakistan. The study results designate that residents believe that CPEC infrastructure projects will significantly improve residents’ life quality through more job openings and community poverty reduction. Still, they raised their concerns regarding environmental protection issues in the region. The findings specified that residents had an optimistic approach to better educational productivity by adopting environment-oriented policies. Policymakers should establish new CPEC study centers in different areas, and investors should be encouraged to participate in the industrial sector. Officials can overwhelm community worries about environmental degradation. Government officials in both countries can utilize the findings to raise public awareness about CPEC’s social, economic, cultural, mental wellbeing, and ecological implications.

## Introduction

The goal of sustainable development has become a focal point worldwide due to its positive influence on health, quality of life, environmental sustainability, and economic progress (Ahmed et al., 2017; Fu and Abbas, 2021). The policymakers have strongly emphasized various criteria to achieve these sustainable development goals (SDG) that influence the community’s wellbeing (Abbas et al., 2021; Li et al., 2022; Zhou et al., 2022). Officials have placed a strong focus on various measures for economic prosperity in the region (Aman et al., 2019; Li et al., 2022). Regardless of their status, many countries have established different policies and development plans to achieve the SDGs, such as property rental value and sustainable urban planning (Abid and Ashfaq, 2015; Mamirkulova et al., 2020; Hussain et al., 2021). Similarly, China and Pakistan designed an economic giant project that would last a long time. For instance, it has provided opportunities for competitive firms’ performance under CPEC projects in the region (Abbas et al., 2019b; Mubeen et al., 2020; Wang et al., 2021). It would benefit both economies as a bilateral initiative for regional development. The “China Pakistan Economic Corridor” (CPEC) symbolizes regional cooperation. It is economic cooperation based on multi-projects initiatives that aim at assisting local inhabitants while also advancing both countries’ economies (Ahmed and Mustafa, 2016).

Researchers have mostly ignored the cultural, educational, social, environmental, and economic implications of the CPEC megaprojects, particularly when considering all stakeholders, including the general public, legislators, financial institutions, and the media (Abbas et al., 2019a; Alam et al., 2019; Hussain et al., 2019; Abbasi et al., 2021b; Azadi et al., 2021; Lebni et al., 2021). Few research studies looked at this mega project’s educational, social, environmental, health, and economic issues in Pakistan amid the COVID-19 crisis (Abbasi et al., 2021a; Aqeel et al., 2021; Su et al., 2021a,b). The CPEC has initiated serval projects to boost China-Pakistan cooperation to strengthen their economies by promoting free trade zones. Even though CPEC is still in its infancy, policymakers and government officials believe it would be a “game-changer” for both countries. It has the potential for countless commercial and employment possibilities for the local community, residents, and foreign communities. There are numerous grounds for proposing domestic and global infrastructure development projects to foster economic growth in South Asia, including the region’s low resources, particularly in community development and connecting emerging countries’ economic ventures to diverse financial hubs and global markets. Besides, development gaps between the developed and developing countries are still uncovered (Bhattacharyay et al., 2012; Kanwal et al., 2019; Latif et al., 2020).

The China–Pakistan Economic Corridor (CPEC) project is significant for China and Pakistan, with good regional cooperation and economic prosperity to improve health, education, and environment (Pouresmaeil et al., 2019; Fattahi et al., 2020; Azizi et al., 2021). It will benefit Pakistan, China, India, and Iran for the local communities’ mental and economic wellbeing even amid COVID-19 challenges (Moradi et al., 2020; NeJhaddadgar et al., 2020; Maqsood et al., 2021; Rahmat et al., 2021). This project is also helpful for the entire international community (Kanwal et al., 2019; Latif et al., 2020; Pitafi et al., 2020). China has made significant investments in the CPEC, one of the most important foreign investments in the country’s history, as part of the “One Belt, One Road” plan (Younis et al., 2020; Islam et al., 2021a; Pitafi and Ren, 2021).

Pakistan is currently dealing with many social, economic, and environmental issues (Anser et al., 2020; Islam et al., 2021c,d; Wu et al., 2021). The prominent issues are poverty, inadequate schooling, infrastructure, security threats, and worst unemployment conditions (Siddiqi et al., 2019; Akhtar et al., 2021b; Islam et al., 2021d). According to officials from both countries, Pakistan will solve its problems if CPEC programs run effectively. On the other hand, China will broaden its influence, strengthen its global presence and secure potential oil and trade routes (Makhdoom et al., 2018). The CPEC is a multidimensional economic initiative to improve local connections between China and Pakistan and between China and Europe. Road networks, power, manufacturing, industries, and other development initiatives are all part of it (Malik, 2017). Policymakers in China have concentrated their efforts on boosting the economy, setting new financial goals, investigating global new markets, and seeking investment opportunities (Abas et al., 2017; Akhtar et al., 2019; Siddiqi and Akhtar, 2020). The Chinese government has established the One Belt One Road (OBOR) megaprojects to attain this goal. This project includes the CPEC, regarded as a game-changer for Pakistan’s economy (Sheu and Kundu, 2018).

This study aims to illuminate the social, economic, and environmental elements of Pakistan’s CPEC development. Additionally, to ascertain neighborhood residents’ impressions of this mega project’s scale. Further, this research tries to debunk fallacies perpetuated by Indian media in the public consciousness. This research study has incorporated three basic sustainability dimensions—economic, environmental, and social—to explore sustainable development in Pakistan. This study provides a scientific report on Pakistanis’ community perceptions of the CPEC as a game-changer. This research plan shows how understudy variables like poverty reduction, quality of life, work opportunities, educational growth, and environmental monitoring can help the CPEC mega project from the initial stage to completion. According to this study’s central assumptions, the China–Pakistan Economic Corridor provides opportunities to improve the local community members (Hadi et al., 2018). This mega project of CPEC is a combination of several schemes that involve healthy economic and social growth of different sectors of Pakistan. An integrative understanding is needed to integrate empirical research into local and regional development through CPEC.

Any country’s economic, environmental, and social concerns are the most important SDGs. Community expectations and perspectives on CPEC megaprojects are a significant issue in today’s environment because informed consent from local stakeholders will help policymakers achieve their objectives. As a result of the study’s findings, Residents may support CPEC megaprojects, which offer job opportunities, a road and rail network, local community high-standard quality of living, and poverty reduction. This paper suggests that the government invest in new educational institutions and let businesses play their vital role in making investments in the industrial sector to develop environmental regulations to maximize the benefits derived through CPEC megaprojects (Philip and Iorember, 2017; Goshit and Iorember, 2020; Goshit et al., 2020; Jelilov et al., 2020). Policymakers, specialists, and academic researchers will profit from this study (Usman et al., 2019; Dabwor et al., 2020; Iorember et al., 2020). As a result, the proposed study methodology establishes an integrated framework for assessing the CPEC’s favorable image in Pakistan regarding the quality of life, job possibilities, poverty reduction, educational development, and environmental protection measures (Iorember and Jelilov, 2018; Iorember et al., 2019; Usman et al., 2020). Government officials and legislators should raise public understanding of CPEC’s activities and advantages to gather support (Iorember et al., 2021).

Furthermore, elected officials can learn about people’s impressions of initiatives and projected advantages, allowing them to make better investment decisions and choose projects that deliver the most social policy benefits for the least amount of money. According to the social exchange theory, local inhabitants are more inclined to support reciprocation if they see beneficial outcomes from services. During the exchange, not only current advantages are examined, but also future benefits. By incorporating local populations through awareness campaigns, the findings of this project will help both China and Pakistan inadequately carry out CPEC operational activities (Haider and Waqar, 2019). This study can also help aid communities in China and Pakistan due to the CPEC. Both countries’ achievements could be crucial in achieving the SDGs.

The social exchange hypothesis provides a theoretical basis for the investigation. The SET, which plays a crucial part in driving primary orientations, postulates that social interactions result from mutual benefits, where the benefits are expected to exceed the project’s expenses. Socio-economic wellbeing is a process two-way’s win-win situation, and both countries anticipate mutual benefits that help reduce payments. According to social exchange theory, human ties are strengthened in the presence of rewards and weakened in the absence of rewards. Suppose the residents of local communities believe that CPEC developmental schemes are advantageous for the region to boost economic, social, cultural, and environmental benefits. In that case, they will actively support the ongoing projects and vice versa. The greater the advantages of the CPEC economic projects, the stronger the local population’s support for its successful running operations. While numerous researchers have applied the social exchange theory in various contexts, it has little significance for assessing widespread acceptance and approval for multinational corporations. This study subsidizes the body of information by analyzing social interactions and the benefits that the local community would gain from the implications of the CPEC projects.

## Literature Review

There are just a few kinds of research on the effects of CPEC on the Pakistani community. This research involved a thorough examination of the past literature in two fields. First, this study focused on the existing literature and attempted to identify the study’s literature gap.

### Economic Corridors

Economic corridors are considered similar to transportation corridors. A transportation corridor is a system that connects financial hubs within or across countries (Hao et al., 2020). As these corridors are expanded to incorporate other states, investment and multilateral commerce will increase. Maintaining and expanding such transportation networks, on the other hand, involves a significant investment of time and resources. As a result, an Economic Corridor is constructed as a transportation corridor with the primary goal of infrastructure improvement (Tong, 2014). Economic corridors are cross borders for international product and service demand and supply. There are no hard and fast rules for identifying an economic corridor since each is unique in location, execution, and duration (Sheu and Kundu, 2018). There are four distinct progressive stages in an economic corridor, each combined into the next using a more radical approach. Typically, storage and transportation come first, followed by logistic corridors (Schimmel et al., 2007). As a result, the transportation corridor is a base for developing later-stage corridors. A trade corridor contributes to creating an industrial corridor, which stimulates economic growth (Raza et al., 2018). Pakistan and China have friendly ties because they share four issues: geo-strategic concerns, energy security concerns, economic cooperation, and security concerns (Rahman and Shurong, 2017).

Pakistan’s unemployment rate continues to fall every day due to population expansion and a wealth of untapped natural resources, all of which contribute to poverty, malnutrition, and social marginalization. During these trying times, the CPEC may prove to be a godsend for job creation and long-term, inclusive economic growth in the region and Pakistan. Previous studies have established that the CPEC projects help create revenue and help construct regional and local economic zones to boost travel and tourism development, benefiting the local community and influencing residents’ attitudes toward the project’s success.

### The China-Pakistan Economic Corridor

Since China announced its official involvement in Pakistan in April 2015, a frequent theme in the literature has been the economic benefits of connecting Gwadar and Xinjiang (Zhang et al., 2017, 2018; Downing et al., 2021; Mamirkulova et al., 2022). According to previous records, the relationship between China and Pakistan strengthened in all areas from the 1970s (Zhang et al., 2017, 2018; Downing et al., 2021; Mamirkulova et al., 2022). It was partly due to the two countries’ leaders having similar philosophies. Similarly, it was discovered that China generously sponsored Pakistan’s nuclear, missile, military, and economic sectors when the US imposed sanctions (Nabi et al., 2018). This study offers valuable results for policymakers’ trust in forging closer relations between Pakistan and China. As a result of their close friendship, the CPEC has become a significant accomplishment (Hadi et al., 2018). China has been attempting to reclaim its former glory for decades (Malik, 2018). China is developing a leading position in Asia and worldwide for political, social, and economic cooperation through the Belt and Road Initiative (Malik, 2017). China began by forming alliances with a small number of non-allies before gradually widening its sphere of influence (Stern, 2001; Ramay, 2016). China has also held a neutral position in foreign affairs, focusing mainly on economic growth (Makhdoom et al., 2018).

President Xi laid the groundwork for it by establishing the “Constructive Engagement” program. As a result, a strong emphasis on economic engagement was placed on improving the favorable policy of naval bases and the Development Bank, among other countries (Khetran and Saeed, 2017). Compared to the current monetarist system and the United States’ dominance in the international financial sector, the Development Bank and Asian Infrastructure Creation are modest (Hussain and Hussain, 2017). The String of Pearls, a network of seaports in Burma, Bangladesh, Pakistan, and Sri Lanka, is also a major strategic initiative to contain India (Hao et al., 2020). “The enemy’s enemy is your comrade,” as the saying goes. On the other hand, China is forging forward, with the CPEC serving as a strategic transportation route. It has become one of the most contentious issues on both a national and international level (Haider and Waqar, 2019).

According to the CPEC, Chinese financing and investment will support Pakistani business industries and SMEs in their operational activities, considered the economy’s backbone (Dhakate and Joshi, 2020). As previously stated, the CPEC will empower rural residents to start a local firm on a shoestring budget (Chen et al., 2018). Many people in rural areas cannot begin businesses as they lack financial resources. Besides, less market demand is another challenge for their products or services (Akhtar et al., 2021a). The CPEC will assist them and foster the entrepreneurial goals of rural Pakistanis (Butt and Butt, 2015). The CPEC can significantly predict economic growth in both countries (Bhattacharyay et al., 2012). China’s investment in the energy industry and infrastructure has already expanded due to the CPEC’s completion, with more expected in the future, recognizing the CPEC’s critical role in bolstering several industrial sectors. This influx of cash will, in turn, increase Pakistan’s economic growth and economic trend. For example, the CPEC was said to have expanded public and private infrastructure investment, which is crucial for economic growth (Ali et al., 2018).

The CPEC has increased investment in various areas, such as energy issues, transportation facilities, oil and gas direct, and indirect contribution to regional and local economic growth (Ali, 2018). The CPEC will also boost regional collaboration and trade between the two countries and other South Asian countries (Jiang et al., 2021; Zhang J. et al., 2021). As a result, it is expected that individuals in China and Pakistan will have sufficient resources, assisting in economic growth and poverty reduction (Ali, 2018). The China-Pakistan Economic corridor (CPEC) would promote development in various sectors, including business and non-business, in Pakistan’s rural and urban areas (Alam et al., 2019; Shi et al., 2021). On the other hand, this will help Pakistan’s economic development by allowing local communities to start enterprises or find work, resulting in a more favorable public opinion of these initiatives (Guoqing et al., 2021). The dynamic depicts the high mobility of social risk in the mining industry and the wide range of initiating or impacted parties, boundaries, and conditions that can be engaged (Peng et al., 2019). Many Asian countries contend with the complexities and inconsistencies in their legal frameworks to resettlement demands and increasing requests to safeguard displaced persons (Guoqing et al., 2021). China’s knowledge and innovation have combined a practical focus on adapting what is appropriate and developing indigenous abilities and instruments with a willingness to learn from global experience (Peng et al., 2019). According to the neoclassical growth theory, resource endowment and infrastructure are the most explanatory elements in rural development (Wang et al., 2020; Jiang et al., 2021). A country’s energy system has a complex impact on its economy. A decrease in energy supply has a dampening effect on economic activity (Zhang R. et al., 2021).

Multiple studies have proved the CPEC’s numerous benefits to society, including expanded access to markets, educational networks, and social interactions, the bridging of social divides and prejudice, and, most importantly, the easing of social exclusion (Wang et al., 2020). China’s economic and commercial invasion will turn the entire community, mainly rural areas, into a commercial and social hub. These accomplishments are the outcome of societal breakthroughs, medical advances, and the growth of smart cities and towns (see Figure 1).

**FIGURE 1:** Proposed model.

### Hypothesis

H1. The CPEC development will significantly influence the Pakistani local community’s quality of life.

H2. The development of the CPEC projects would significantly influence Pakistanis’ community perception to create more job opportunities.

H3. The CPEC megaprojects will considerably help reduce poverty among the local community in Pakistan.

H4. The CPEC development would create more educational opportunities for the local community.

H5. The CPEC economic development projects would raise community concerns on environmental security in Pakistan.

#### Research Methodology

This study aimed to examine prior literature to determine the Impact of CPEC projects on the Pakistani population. As a result, to fully comprehend this issue, we review the past research in high-quality academic publications and books (Khan et al., 2020; Islam et al., 2021b; Lai et al., 2021). As a consequence of our study, 27 essential rudiments of the CPEC project have been identified. We also conducted a survey to learn about the local community’s perceptions of the China-Pakistan economic corridor. We discussed 16 professionals before conducting the study to guarantee a sufficient and correct model. A survey and interviews were used in this research project (mixed-method).

### Conceptual Model

PLS-SEM is a multivariate analysis technique that is especially effective in the social sciences because it generates structural equation models based on variance (Rigdon, 2016). A path model that incorporates latent constructs includes a measurement model that elucidates the links between the latent variables and the path model’s indicators. The SEM method is frequently used to examine and test complex connections and causal linkages systems (Rönkkö et al., 2016; Rigdon et al., 2017). SEM is a statistical technique that combines regression, multiple correlations, factor analysis, and path analysis techniques. The conceptual model is defined as the links between latent variables and the observable variables that correspond to them. Because latent (unobserved) variables cannot be measured directly using manifest (observable) variables, it is critical to create a model to quantify them. According to this study, the model developed is based on 24 observed variables based on the development of the CPEC. These variables, which are referred to as exogenous latent variables, are divided into five categories: the quality of the local community, job opportunities, poverty reduction, educational advancements, and education (Krajangsri and Pongpeng, 2017).

### Research Design, Sample, and Data

The purpose of this study was to demonstrate the value of the CPEC from the perspective of local populations in terms of environmental protection, improving quality of life, expanding educational and employment opportunities, and alleviating poverty, and improving market growth in the region. The study used a mixed-methodology approach to test the hypotheses by testing the empirical data (Local Burden of Disease, 2021; Paulson et al., 2021). The information is gathered through a standardized survey and interviews with Pakistanis who live in different areas of Pakistan, where the CPEC route crosses. The questionnaire was written in English for Pakistanis to understand what it was asking. We did, however, offer assistance to those who were having difficulty deciphering the questions. The survey form contained two sections. Age, education, and gender were all covered in the first section; on the other hand, the second section concentrated on the key variables and their corresponding information. The investigators recruited respondents across all provinces in Pakistan to increase the effectiveness of the survey. This study invited respondents who were currently finishing or closer to completing CPEC projects. In addition, we looked at well-educated respondents, as less educated people are less likely to be familiar with CPEC and its services.

The researchers distributed five hundred surveys to the respondents and received satisfactory results. English, widely spoken as a second language in Pakistan, was this survey’s polling language, and respondents generally favor it. The investigators assisted responders in identifying points of argument. The survey selected this sector because the less educated population frequently faces difficulty completing survey questionnaire forms. They might be unaware of CPEC operations. This research aids government officials in defining their aims while informing the public about the importance of the CPEC. We collected and submitted all data over three months and received 523 survey responses. The investigators omitted twenty-eight incomplete questionnaire forms. As a result, this study could only analyze and validate the model through the valid responses of 459 respondents.

Table 1 indicates an overview of the respondents who completed the questionnaire. The survey received responses from 310 men (67.53%) and 149 women (32.46%). This survey incorporated the collected data from respondents aged 25 or above. It was helpful to predict CPEC projects’ benefits precisely. The investigators classified respondents into five groups based on their actual age.

**TABLE 1:** Respondents’ profile.

Respondent description	Frequency	Percentage
Male	310	67.53%
Female	149	32.46%
	**Age of respondent**	
25–30	150	32.67%
31–35	250	54.46%
36–40	59	12.85%
	**Educational details**	
Bachelors	300	65.35%
Master	159	34.64%

### Sample

This paper incorporated the convenient sampling technique for desired data collection from recruited participants of five major cities of Pakistan. The research was limited to 459 respondents who completed the questionnaire entirely. The participants in this study were both males and females ranging in age from 25 to 45 years, with the average age being 25 years. This survey mainly focused on evaluating the development of the CPEC and its dimensions in forecasting the growth of the projects. The researchers devised a comprehensive strategy and conducted a thorough literature review concerning the proposed study. The study formulated the hypothetical comprehension of the subject under consideration in the first step. Thus, the investigators performed extensive literature reviews by focusing on published content in high-quality journals and books and aligned it with research questions. The researchers used Smart PLS version 3.4. Software programs measure the validity and precision of the received data and find it accurate.

#### Data Analysis

This analysis reports on the detailed results derived from empirical data provided by the study participants. In structural equation modeling, PLS-SEM is a helpful tool to derive results for this type of research. The investigators applied the PLS-SEM method for data analysis. Table 2 reveals the results of this analysis. This study’s main focus was to assess the progress of the CPEC for regional development (Gudergan et al., 2008; Hair J. et al., 2017). There are two kinds of evaluations: the first is the evaluation of the measurements of the external model, and the second is the evaluation of the internal structural model. The model was investigated and validated using Smart-PLS software.

**TABLE 2:** Mean scores (M), standard deviations, values of Kurtosis, and Skewness.

Items	Mean	*SD*	Kurtosis	Skewness
QOLC1	5.000	1.501	–1.026	–0.722
QOLC2	5.000	1.526	–1.268	–0.572
QOLC3	5.000	1.426	–0.939	–0.698
QOLC4	5.000	1.473	–1.413	–0.213
QOLC5	5.000	1.441	–1.101	–0.574
OFJ1	5.000	1.451	–1.131	–0.545
OFJ2	5.000	1.529	–1.335	–1.335
OFJ3	5.000	1.556	–1.456	–0.317
OFJ4	5.000	1.501	–1.026	–0.722
OFJ5	5.000	1.354	–0.465	–0.944
OFJ6	5.000	1.449	–0.893	–0.765
ROP1	5.000	1.405	–0.725	–0.827
ROP2	5.000	1.391	–0.534	–0.898
ROP3	5.000	1.426	–0.939	–0.698
ROP4	5.000	1.457	–1.073	–0.649
ROP5	5.000	1.456	–0.701	–0.879
DOE1	5.000	1.487	–0.799	–0.857
DOE2	5.000	1.418	–0.574	–0.923
DOE3	5.000	1.404	–0.437	–1.001
DOE4	5.000	1.435	–0.635	–0.902
DOE5	5.000	1.526	–1.268	–0.649
SOE1	5.000	1.457	–1.073	–0.879
SOE2	5.000	1.456	–0.701	–0.857
SOE3	5.000	1.487	–0.799	–0.722
DOCP1	5.000	1.501	–1.026	–0.572
DOCP2	5.000	1.526	–1.268	0.000
DOCP3	5.000	1.426	–0.939	–0.698
DOCP4	5.000	1.487	–0.799	–0.857

Table 2 provides an all-inclusive descriptive statistical analysis description, including the mean scores (M), standard deviation scores (SD), Skewness, and kurtosis values. The values in Table 2 revealed that the data of this population produced decent results. See Figure 2 that shows the algorithm model and Figure 3 shows the measurement model (PLS-SEM algorithm). Estimations of structural equations model graphical representation of construct validity and reliability. Graphical presentation of Cronbach’s alpha, composite reliability (CR), and average variance extracted (AVE). The data has shown a normal distribution and supported the outcomes based on statistical analysis (see Table 2).

**FIGURE 2:** Algorithm model.

**FIGURE 3:** Measurement model (PLS-SEM algorithm). Estimations of structural equations model graphical representation of construct validity and reliability. Graphical presentation of Cronbach’s alpha, composite reliability (CR), and average variance extracted (AVE).

#### Evaluation of Outer Measurement Model

A consistency and validity measurement model is being developed to serve as an external measurement model for the observed variables. Conversely, the variables are evaluated using convergent and discriminant validity (Hair et al., 2020). Individual manifest and concept reliability tests are used to assess internal consistency, while convergent and discriminant validity tests determine the variables’ validity (Hair et al., 2012a). Thus, single manifest reliability designates the manifest compared to a latent variable, and it measures consistent outer loadings of the manifest variables. It is acceptable to have a manifest variable value greater than 0.7 when the external loading is more significant than 0.70 (Henseler et al., 2009; Sarstedt et al., 2017). Cronbach’s alpha, composite reliability (CR) scores, and average variance extracted from the measured constructs are some of the tests that can be used in PLS path modeling in determining the convergent validity of the measured constructs (AVE) (Shanmugapriya and Subramanian, 2015; Aman et al., 2021). This study developed a measurement model according to the previously established analysis rules. The reliability and validity tests results are presented in Table 3 and further discussed below. As shown in Table 3, individual construct reliability values are more significant than 0.70 (Ringle et al., 2009). The average reliability value (AVE) for all constructs is greater than the critical value of 0.5, indicating decent reliability (Vinzi et al., 2010; Henseler et al., 2016). Besides, the loadings of all the variables are within the acceptable range. It must reflect values greater than 0.7 for each of them individually. As a result of these findings, the measurement model appears to have sufficient reliability and validity characteristics (Hair J. F. et al., 2017; see Figure 2 and Table 3).

**TABLE 3:** The measurement model displays a convergent validity, alpha (_), and reliability.

Construct	Items	Loadings	Cranach’s alpha	CR	Ave
Implementation of CPEC	CPD_1	0.885	0.905	0.933	0.778
	CPD_2	0.867			
	CPD_3	0.869			
	CPD_4	0.906			
Quality of local community	COLC_1	0.847	0.892	0.963	0.839
	COLC_2	0.847			
	COLC_3	0.795			
	COLC_4	0.791			
	COLC_5	0.893			
Stability of environment	SOE_1	0.908	0.808	0.920	0.698
	SOE_2	0.925			
	SOE_3	0.924			
Reduction of poverty	ROP_1	0.885	0.939	0.942	0.845
	ROP_2	0.915			
	ROP_3	0.868			
	ROP_4	0.888			
	ROP_5	0.925			
Opportunities for jobs	OFJ_1	0.791	0.894	0.911	0.656
	OFJ_2	0.724			
	OFJ_3	0.762			
	OFJ_4	0.880			
	OFJ_5	0.829			
	OFJ_6	0.863			
Edu. development	DIE_1	0.913	0.952	0.953	0.804
	DIE_2	0.938			
	DIE_3	0.925			
	DIE_4	0.942			
	DIE_5	0.850			

#### Inner Structural Model’s Evaluation Through Smart PLS

It was discovered in this study that the measurement model’s validity and reliability had been evaluated and confirmed. Afterward, we assessed and confirmed the validity and reliability of the measurement model, which served as the final step in the process.

#### Measuring the Value of R2

A measure of the variance explained by endogenous variables and a measure of the predictive accuracy of a model calculated; the R2 statistic can be calculated (Sarstedt et al., 2017). An estimate of the variance explained by endogenous variables and a measure of the predictive accuracy of a model calculated; the R2 statistic can be calculated (Sarstedt et al., 2017). The final model’s R2 indicated that independent factors explained the variance in CPEC implementation among the study’s sample population. The results of this study were as follows: To be considered predictively accurate, according to Keaveny et al. (1997), a model’s R2 should be greater than 0.10 to be considered valid. If the value of R2 is less than this, it is assumed that the conceptual model cannot describe the endogenous variables in the data set.

#### Path Coefficient and T-Statistics

It is possible to obtain a standardized beta coefficient’s path coefficients in a PLS model (β) (Hair et al., 2012b). A unit variation in exogenous variables is equivalent to a possible variation in endogenous variables, and the path coefficient denotes this possibility. The values of each path are used to compare the conceptual models; a higher value indicates a more significant influence on endogenous variables than a lower value. The *t*-test is used to determine the significance of the path coefficient(s) in question. A bootstrapping procedure is used to determine the importance of a hypothesis (Chin, 1998). For statistical significance at the 5% significance level, the t-statistics values must be equal to or greater than the cutoff value of 1.96 (Hair et al., 2012a). See Table 4 for testing proposed hypotheses.

**TABLE 4:** Hypothesis testing.

Hypothesized path	t-statistics	*p-*value	Decision
Quality of local community > CD	145.23	0.000	Supported
Opportunity for job > CD	163.24	0.000	Supported
Reduction of poverty > CD	205.12	0.000	Supported
Stability of the environment > CD	269.45	0.000	Supported
Development in education > CD	283.32	0.000	Supported

Table 4 results specified that the findings had verified the proposed hypotheses. Therefore, the proposed hypotheses of variables in this study significantly affect the development of CPEC is accepted and proven (see Figure 4).

**FIGURE 4:** Structural model of this study (the analysis based on PLS-SEM bootstrapping).

#### Effect Size of the Model

According to Cohen, a strong effect is observed at a value of 0.35. A moderate effect occurs at 0.15. It indicated a weak impact occurs at 0.02 (Goodhue et al., 2006). The values calculated using the PLS-SEM technique are presented in Table 5 (Henseler and Fassott, 2010). As shown in Table 5, results (f2) reveal the magnitude of the effect and the good relationships among the understudied variables. Table 5 summarizes the findings of this study’s analysis.

**TABLE 5:** Effect size.

Exogenous latent variables	Effect size *f*2	Total effect
Quality of local community > CD	12.81	High effect
Opportunity for job > CD	7.78	High effect
Reduction of poverty > CD	10.13	High effect
Stability of the environment > CD	8.65	High effect
Development in education > CD	12.92	High effect

#### Model Predictive Relevance Q2

It is necessary to evaluate the quality of the smart PLS path model using the predictive relevancy model. It is hypothesized by the Predictive Relevance Model (Q2) that the proposed model may be capable of predicting the endogenous latent constructs that were discovered in this study. When using the smart PLS-SEM, the predictive relevance (Q2) must value calculated in the model be (> 0) greater than zero for the specific endogenous latent construct under consideration.

Figure 5 shows a decent value for this particular model’s predictive relevance (Q2); this value exceeds that of the predictive relevance’s upper limit for the model. These findings provide additional support for the predictive model relevance of the path model, which is appropriate for the endogenous constructs under consideration (see Figure 5).

**FIGURE 5:** Assessment of inner structural model.

The strategies used to analyze the structural model’s results are as follows: thus, the effectiveness of the model prediction abilities and the relationship between the components must be considered. The (R2) coefficient of determination based on endogenous latent variables, the vital assessment criterion for an inner structural model, helps to believe it. Other practical ways for analyzing the internal structural model, in addition to the path coefficient and t-statistic value, included effect size (f2), the goodness of fit (GoF), and the model’s predictive relevance (Q2).

#### Standardized Root Mean Square Residual Index—Standardized Root Mean Square Residual

The standardized root mean square residual (SRMR) index in statistics compares the standardized residuals between the hypothesized and observed covariance matrices (Henseler and Fassott, 2010). Model fit is a metric that measures the relationship between a projected and estimated designed model fit in a given situation. As long as the SRMR is equal to or less than 0.08, it suggests adequate performance, fit, and research model; all of these features are regarded as positive signs (Pavlov et al., 2021). As shown in Table 6, the results show that the SRMR value is 0.073. It means that the model is a good match. The value of the Chi-Square (_2) is 1665.878, and the NFI shows a value of 0.772 in Table 6.

**TABLE 6:** Model fit summary.

SRMR	Estimated model
d_ULS	0.078
D_G1	2.447
D_G2	0.564
Chi-square (_2)	444.34
NFI	0.923

#### Perceptions of the China-Pakistan Economic Corridor Projects’ Impact on Pakistani Community’s Long-Term Development

##### Interview Results

We interviewed 35 community representatives to acquire a fair and informed opinion about the value of CPEC projects for the Pakistani community concerns the sustainable growth of CPEC. This chapter analyses the judgments of these professional interviewers on the influence of society. Almost 75% of the community expert indicated that CPEC displays a vital function in Pakistan’s community development. In comparison, 25% of experts suggested that although they prefer CPEC for the Pakistani community, they are scared of external dangers to CPEC. Significantly they highlighted their concern about the role in developing this large enterprise. These findings offer a significant indicator of the relevance of CPEC for the interests of both governments.

## Discussion

The findings indicate that the development of CPEC has been examined from two perspectives. Social objectives include a good standard of life, employment opportunities, poverty reeducation, and two additional purposes: educational advancement and environmental protection. The pandemic has caused mental wellbeing issues and affected individuals quality of life (Aqeel et al., 2022). From a community perspective, it was decided to evaluate CPEC projects based on their perceived ecological health, quality of life, educational possibilities, and poverty reduction. As a result, we collected data from inhabitants of Pakistani communities whose social and economic prospects may be adversely affected by CPEC development. According to our results, the Pakistani public believes the CPEC would spur economic growth. Our findings corroborate prior research suggesting the project will generate jobs, businesses, trade, services, and other commercial activities that will benefit the country economically. Additionally, the social implications are favorable, indicating that the new adjustments to the global project would help the local community adapt to them.

It is the first time empirical data gathered from Pakistanis living in areas where CPEC projects are tested (Abid and Ashfaq, 2015). In an attempt to determine the significance of CPEC in terms of economic growth, poverty reduction, and environmental protection, the authors relied solely on qualitative data gathered through interviews to arrive at their conclusions. As a result, the research findings are precious in theoretical contributions and practical implications. Several social exchange theories have been proposed (Cook et al., 2013). The support of local communities for policy is more likely to occur if they believe it will benefit them; otherwise, they are more likely to be opposed. As a result, we put the model to the test and discovered that local communities believe CPEC provides numerous benefits and intend to support its expansion. According to this report, residents were concerned that the CPEC project would harm the environment and opposed it. During the development stage, the construction of roads and transportation infrastructure has an unavoidable effect on the people’s quality of life along these roads and infrastructure. Because of a lack of greenery and more severe weather in sandy areas, the CPEC’s major routes significantly impact people’s livelihoods, particularly during the summer months, particularly in China’s provinces. So they have a negative attitude toward the environment; however, environmental protection agencies should protect and safeguard the environment from any adverse effects of these business ventures. As a result of the information-sharing programs offered by these organizations, residents should be aware of potential environmental threats and mitigation measures that may be implemented.

According to Amir (2016), While the CPEC does not adequately protect the region’s ecosystem from pollution, it would still result in a slew of environmental problems even if it did. According to Mehmood-ul-Hassan (2016), Local communities face various challenges regarding construction and new construction. These challenges can negatively impact their daily lives. Our research revealed that putting the CPEC into effect would significantly improve the overall quality of life for citizens in the region. As Khan and Khalid (2018) discussed, people can earn more money by participating in new projects while also gaining new experiences and improving their living conditions, as previously stated.

Similarly, Lee et al. (2018) asserted that the construction of the CPEC would significantly improve the quality of life for the average person of Pakistan. It appears that they do not believe the CPEC will strengthen their educational standards, based on our findings. Interestingly, our research revealed some unexpected results in terms of the level of academic quality. On the other hand, CPEC has not announced any educational programs or taken part in discussions about educational policy reform as of this writing. It has resulted in them having low expectations of their abilities in terms of academic achievement. However, many Pakistanis study at Chinese universities, but they do not believe that the CPEC prioritizes Pakistan’s educational infrastructure. CPEC’s expansion, according to the findings of this study, is expected to result in a significant increase in employment opportunities for the general public. Programs that are cutting-edge and make use of global resources are available. According to Hansen et al., citizens have new opportunities to improve their lives.

A past study Ullah et al. (2018) has predicted that the CPEC will significantly increase the number of job opportunities for Pakistan’s local communities and the general public. According to Ali et al. (2018), the CPEC is a megaproject that will generate millions of jobs across a wide range of industries (Javaid and Javaid, 2016), were correct in questioning whether the CPEC would make finding work more accessible. People believe that job opportunities (such as those created by the CPEC) will alleviate poverty. As a result, the CPEC can be a powerful predictor of poverty. Locals anticipate a slew of job openings, many of which will be high-paying jobs that will enable them to escape poverty due to CPEC. Wolf (2020) reports various CEPC benefits, including employment opportunities, poverty reeducation, and social welfare, consistent with our findings.

### Implications for Practices

The study’s findings have significant consequences for Pakistani politicians and residents and Chinese citizens in general. According to this article, the expansion of CPEC has altered residents’ perceptions of normalcy, employment opportunities, and low poverty due to their economy’s reorganization. The vast majority of citizens are in favor of the CPEC. As a result, they will help shape the future of the CPEC’s potential benefits. Residents believe that the city’s overall quality of life may have several advantages. People should obtain psychological counseling to enhance their overall quality of life. Pakistan’s government must develop policies that priorities senior folks’ health and wellbeing.

The government should encourage the development of CPEC megaprojects to improve the efficiency of operating activities in the regions. The education of the general public about the CPEC projects and their benefits is a top priority for government officials in the country’s capital. This strategy will have a significant positive impact on the CPEC and other megaprojects in the region. The results of our research revealed that citizens’ perceptions of environmental security are unsatisfactory, as demonstrated by our findings. The CPEC project is currently underway, and the infrastructure for the associated areas is being built. Their point of view has shifted because of the difficulties and obstacles associated with the CPEC roads. China and Pakistan should prioritize environmental conservation and green practices to make their respective countries more welcoming to visitors and residents from other countries. Their health and safety must be protected at all times, and they must also work to reduce emissions in their respective neighborhoods. Pakistan’s environmental policies are woefully insufficient, implemented in private and public sectors. The Pakistani government must develop written procedures for environmental conservation to gain the local population’s attention. We discovered that many individuals hold negative attitudes toward education, which the CPEC can help change through its implementation. Whether the CPEC is a good indicator of high-quality rural education is a contention between the two. It sends out alarming signals to the governments of China and Pakistan, urging them to launch regional educational and awareness campaigns as soon as possible to address the situation.

According to the World Bank, the government of Pakistan must build new schools and universities in rural areas. The construction of new schools and colleges, similar to megaprojects that boost economic development and create job opportunities, could benefit people because travel distance is a significant barrier to obtaining an education. Apart from that, government officials in both China and Pakistan should emphasize megaprojects that will improve the quality of life while also creating employment opportunities in the affected areas of both countries. In rural Pakistan, as is the case throughout the rest of the country, many people live in poverty. The government should implement individual benefits and work quotas to assist rural areas in escaping poverty. This study’s authors make several vital policies, and government implications for the future based on empirical evidence gathered during the research. According to our study, policymakers can use the CPEC to assist societies in achieving their social objectives. The final point to consider is how the CPEC can assist communities in achieving their social goals through economic development. An evidence-based questionnaire administered to 495 people (323 men and 122 women) revealed that educated sections of the Pakistani public believe that the CPEC will bring benefits such as improved quality of life, increased job opportunities, and poverty reduction to the country. It will not have any beneficial effects in areas such as the environment or education (Ge et al., 2021).

On the other hand, no statistically significant results were discovered to improve environmental conservation or educational quality. For the CPEC to be fully realized, policymakers should establish new educational institutions, encourage investors to invest in the industrial sector, and communicate environmental strategies. As a result, and in light of the widespread opposition to these projects among the general public, the government should concentrate its efforts on two major initiatives: environmental protection and educational outreach. So the government must come up with more effective policies to provide the general public with sufficient convenience. A strong emphasis is placed on environmental strategies in light of the evidence gathered through the questionnaire and interview, which indicates that the evidence is not supporting perceived ecological conservation. Aspects of quality of life should be considered by policymakers, as many of those interviewed do not believe that the China-Pakistan Economic Corridor will provide them with a high-quality life. Government officials and politicians are also urged to raise public awareness of the CPEC projects and their benefits in their respective communities to garner support from the general public. Overall, the findings of this study strongly suggest that policies be put in place to ensure that the CPEC is used effectively to achieve social objectives.

The CPEC is the core project of the Belt and Road Initiative, which is undoubtedly a key and significant task for Pakistan, China, and the world. Several flaws in the authors’ analysis have been pointed out that these flaws can be seen as opportunities for future research in the field. As a result of this research, several significant factors that can influence the willingness of the local community to support the project have been identified, and these factors are discussed in greater detail below. It is difficult to generalize the findings of this study to the entire population of interest because of convenience sampling in the research. Policymakers should exercise caution when interpreting the study’s findings, considering the study’s context and usability. The information in the present report was gathered through self-reporting, and the results were used to compile the report as it is now. According to the authors, the findings on the media effect can be used to improve strategic communication about the CPEC and local communities and increase public trust in the Belt and Road Initiative. The CPEC project’s progress could be examined in more detail in future research, including determining whether print media, social media, or electronic media all impact the project’s overall success or failure. A prospective research study will address the limitations of this study and the limits of previous research studies. First and foremost, it is noticeable that the study’s sampling scale concentrated on Pakistan’s northwest while neglecting other essential regions such as Pakistan and China, which should be considered. If possible, we strongly advise that data should be gathered from Chinese citizens and residents of other major cities throughout Pakistan to articulate the findings better.

Furthermore, combining data from both samples (Pakistan and China) into a single analysis has the advantage of generating results that are precisely comparable between the two models. For the second time, cross-sectional data has been called out for containing a significant amount of process bias, demonstrated in various studies. Therefore, a large sample size for interviews or longitudinal data collection is recommended for future research studies.

The conversation got interrupted by the arrival of approximately 20 people, most of whom were representatives from various community organizations. We proposed that we look into the viewpoints of less-educated groups on the CPEC to determine whether there were any differences in views among less-educated groups on the CPEC. Thirdly, we underestimated the opinions of male and female residents and those with high and low levels of education and affluence, which opens the door to a new area of research that requires further exploration. Additional testing in Pakistani locations where the CPEC’s lines cross is being done to determine the model’s performance in those locations. According to our research, Pakistanis believe that the advancement of the CPEC has improved their quality of life.

Additionally, they believe that employment opportunities have improved, and people living below the poverty line have decreased. On the other hand, many people regard environmental security and educational excellence as secondary priorities. According to available statistics, numerous researchers have shown interest in working on CPEC projects to evaluate effects on the development of the local community.

## Data Availability Statement

The original contributions presented in the study are included in the article/supplementary material, further inquiries can be directed to the corresponding author/s.

## Author Contributions

All authors listed have made a substantial, direct, and intellectual contribution to the work and approved it for publication.

## Conflict of Interest

The authors declare that the research was conducted in the absence of any commercial or financial relationships that could be construed as a potential conflict of interest.

## Publisher’s Note

All claims expressed in this article are solely those of the authors and do not necessarily represent those of their affiliated organizations, or those of the publisher, the editors and the reviewers. Any product that may be evaluated in this article, or claim that may be made by its manufacturer, is not guaranteed or endorsed by the publisher.
